# Effect of Image Detection and Analysis and Hospice Nurse Mediated Aromatherapy on Pain in Patients with Advanced Cancer in Intelligent Medical Environment

**DOI:** 10.1155/2022/5111021

**Published:** 2022-08-03

**Authors:** Dongmei Shi, YanXia Shi, Ying Li, Jinhua Hong

**Affiliations:** Jiangxi Cancer Hospital, Nanchang 330029, China

## Abstract

**Objective:**

In order to better alleviate the pain symptoms of patients with advanced cancer, this study adopts image detection and analysis and hospice nurse mediated aromatherapy, so as to comprehensively understand the physical condition of patients with advanced cancer and finally implement the nursing scheme of aromatherapy.

**Methods:**

Sixty advanced cancer patients admitted to a tertiary and grade A oncology hospital in Jiangxi Province from December 2020 to March 2022 were selected. This study was randomized into trial and control groups. The control group contained 30 regular treatment patients and 30 regular nursing patients for advanced cancer patients, and the trial group performed a 28-day hospice care specialist nurse-mediated aromatherapy based on the control group. Pain and quality of life scores were measured before and after the intervention in both groups. The experimental group consisted of 30 cases, with the mean age of 58.2 years; the control group consisted of 30 cases, with the mean age of 58.6 years.

**Results:**

60 patients with advanced cancer were selected for group comparison. The results showed that the effect of aromatherapy mediated by hospice nurse on pain score, QLQ-C30, index value of patients with advanced cancer (the experimental group) was better than that of patients with advanced cancer (the control group).

**Conclusion:**

Through retrospective analysis, we investigated the patients with advanced cancer and discussed the difference between conventional therapy and aromatherapy. The results showed that aromatherapy based on image detection and analysis and mediated by Anning nurses was helpful to alleviate the physical function of patients with advanced cancer and improve their quality of life, which provided a reference for clinical application.

## 1. Introduction

With the rapid development of high technologies such as artificial intelligence and sensing technology, smart medicine rises. It is to build a regional medical information platform for health records and use the most advanced Internet of things technology to realize the interaction between patients and medical personnel, as well as between medical institutions and medical equipment, so as to gradually achieve informatization and make the medical service intelligent in the real sense. In the intelligent medical environment, the method based on image detection and analysis has also been widely used in medical treatment. At present, with the increasing global cancer incidence rate, cancer has become the “number one killer” threatening human life and health. The first problem that scientists have not yet solved is the problem of cancer treatment. In particular, patients with advanced cancer suffer from psychological and mental torture in addition to physical pain. It has seriously affected the physical and mental health and quality of life of patients. Previously, most of the patients were relieved by taking drugs. Now, safe and effective nursing methods are encouraged. Aromatherapy can relieve the cancer pain of patients and provide reference for the care of patients with pain. Therefore, Tang et al. pointed out that, due to the disease itself or treatment, cancer patients will be accompanied by physiological, psychological, spiritual, and other symptoms throughout the course of the disease, which seriously affect the quality of life of patients [1]. Aromatherapy is a method of preventing and treating diseases by making fragrant drugs into appropriate dosage forms, so as to act on the whole body or part. It can relieve anxiety and dry skin. In European and American countries, this law has been widely used in the field of hospice care [2]. Therefore, Lin et al. proposed that aromatherapy, as a commonly used complementary medical therapy, is widely used in cancer treatment and palliative care to improve the quality of life of cancer patients, reduce their mental stress, reduce their psychological disorders, alleviate their disease pain, and improve their quality of life [3]. Xu et al. showed that aromatherapy can be better used in clinical nursing of cancer patients in the future from the effects of aromatherapy on sleep, mood, nausea and vomiting, fatigue, pain, edema, constipation, and so on [4]. Xiuqiao et al. also pointed out that the application of aromatherapy is to alleviate the symptoms of nausea and vomiting, so as to alleviate the pain of patients, and can effectively improve the nursing satisfaction of patients. It should be further popularized and applied in clinic [5]. Zhang et al. found through experimental research that aromatherapy is simple and operable for patients with advanced cancer, and its use in hospice care can improve the quality of life of elderly patients with malignant tumors at the end of life, which is worthy of clinical promotion [6]. Wu et al. also concluded through experiments that actively carrying out hospice mediated aromatherapy for advanced cancer patients who have no hope of cure can promote the reduction of their pain experience and the improvement of their quality of life, which is of positive significance [7]. Moreover, Wei et al. said that aromatherapy uses natural plant spices or aromatic essential oils extracted from them, and the essential oils have two-way regulating effects on the human nervous system, digestive system, respiratory system, skin, urinary system, and so forth [8]. Zeng et al. discussed the effect of aromatherapy combined with repeated transcranial magnetic stimulation on the adverse mood and sleep quality of female schizophrenic patients in remission stage. The clinical effect is significant, which can bring reference significance to this study [9]. Through the research on the impact of hospice nurse mediated aromatherapy on the pain of patients with advanced cancer based on image detection and analysis in the intelligent medical environment, from the results of pain score, QLQ-C30, EORTC quality of life measurement, and total health status index value, it is found that the aromatherapy mediated by Anning nurse has a good therapeutic effect on the body, heart, and soul of patients with advanced cancer and provides a good clinical significance.

## 2. Research Background of Aromatherapy

Aromatherapy originated from ancient civilizations such as ancient Egypt and prevailed in Europe in modern times. It can relieve mental stress and improve physical health by using essential oils. In 1928, the French chemist “Gatfersey” first used the name of aromatherapy, and some began to use it in the scientific journal of aromatherapy. By chance, he found that peppermint or lavender oil has special therapeutic power. The essential oil distilled from aromatic plants is used to obtain the integrated curative effect of body, heart, and spirit. It is an adjuvant therapy. Essential oil contains ketones, esters, and other chemical components, which determine its therapeutic characteristics. It can be used by direct inhalation, bathing, and massage to improve anxiety, pain, fatigue, and wound healing. Like drugs, essential oils mainly affect the limbic system of the brain through sniffing and penetrate into the body through the skin, so as to achieve the purpose of treatment. Cancer is one of the main diseases that human beings are difficult to overcome at this stage, and, globally, the number of people living with cancer is still increasing. Long-term radiotherapy and chemotherapy have led to a significant decline in their quality of life. Li et al. found that cancer can bring many uncomfortable symptoms to patients, such as pain, fatigue, anxiety, and fear. Therefore, cancer pain is considered to be one of the most common and fearful symptoms. Therefore, pain treatment is an indispensable and important part of comprehensive treatment of cancer [10]. Chen et al. found through retrospective research that most end-stage patients are accompanied by infiltration, metastasis, and damage to adjacent organs and tissues and often have different degrees of pain symptoms, such as decreased activity tolerance and function, loss of appetite, nausea, and insomnia. The psychological and spiritual manifestations are as follows: anxiety, depression, fear, inattention, and suicidal tendency in severe cases. In terms of social communication, the reduction of social activities, loneliness, and dependence have seriously reduced the quality of life of patients [11]. In terms of clinical treatment, advanced tumors have lost the best period of radical surgery, and aromatherapy mediated by hospice care has become the main treatment. Zhao et al. pointed out that hospice care is centered on the dying patients and their families and carried out in a multidisciplinary cooperation mode, focusing on the best management of painful symptoms. Moreover, hospice care can effectively solve the psychological and physiological problems of patients with end-stage diseases and their families and play a positive role in improving the quality of life of patients in the final stage of life [12]. Wang et al. evaluated the anxiety, depression, and pain degree of each patient by using various scales and pain digital scoring method and concluded that pain management is an important part of hospice care. It can use effective pain management methods for patients, improve patients' understanding of cancer pain, help patients improve pain threshold, and enhance their pain tolerance, so as to reduce patients' pain [13]. Law et al. pointed out that aromatherapy, as a supplementary care method, has a promising application prospect in cancer patients and can be better applied to cancer patients for reference [14]. At the same time, psychological care should be given to patients. Through aromatherapy methods such as diverting attention, psychological suggestion, deep breathing, and local application of peppermint oil or borneol, patients should relax their body and mind as much as possible, reduce the impact of pain, and improve their quality of life.

## 3. Current Situation and Application of Hospice Nurse Mediated Aromatherapy in Patients with Advanced Cancer Based on Image Detection and Analysis

With the increasing refinement of the computer age, image detection extends the idea of edge detection to identify the entire image, usually to judge whether the detected image belongs to an image in the known image database, or infer that the image is most similar to a known image after comprehensive discrimination. Based on image detection and analysis, it is found that the current situation and application of hospice nurse mediated aromatherapy in patients with advanced cancer are reducing pain, which is usually caused by noxious stimulation, accompanied by a feeling of unpleasant emotional experience, and the stimulation can come from the outside and act on the body surface. According to the survey, more than 50% of cancer patients will have cancer pain of different degrees, which will bring serious negative emotions. Severe cancer pain will seriously affect the quality of life of patients. Through the grouping experimental study, the researchers randomly selected cancer patients and then compared them with essential oil massage combined with hospice care, simple massage, and no other special treatment. The results showed that the analgesic effect of essential oil massage combined with hospice care was better than that of other groups, with higher quality of life and less emotional fluctuation. Based on the analysis of the current situation, emotional relief can reduce the generation of negative emotions, which can better illustrate that aromatherapy can be widely used in medicine and has reference significance. Therefore, aromatherapy can be used as one of the adjuvant therapies to control pain. Secondly, aromatherapy can alleviate the nausea and vomiting of cancer patients. Cancer patients will have different degrees of nausea and vomiting after chemotherapy and drug treatment. Some researchers found that inhaling ginger, mint, and lemon compound essential oil and smelling sliced lemon fragrance can effectively alleviate the nausea and vomiting of patients. Therefore, in clinical intervention, we can try to choose the method of aromatic inhalation, combined with essential oil acupoint massage, so as to effectively alleviate the nausea and vomiting of tumor patients. In addition, aromatherapy can relieve the mood of cancer patients. By diverting attention from their own symptoms, cancer patients will not only suffer physical pain but also suffer psychological and mental torture. The intervention of aromatherapy can reduce the physical discomfort of patients. In addition, many cancer patients will have emotional problems such as anxiety and depression, which will affect the quality of life of patients. Studies have found that lavender essential oil has analgesic, anticonvulsant, antidepressant, and sedative effects. In aromatherapy, it is often used to balance emotions and improve anxiety, depression, and other problems and can bring positive effects to patients. Aromatherapy can also improve sleep disorders and improve sleep quality. Sleep disorder is one of the most common symptoms of cancer patients, which can be caused by adverse reactions such as pain, radiotherapy, and chemotherapy, as well as factors such as anxiety and depression. Insomnia can hinder the recovery of cancer patients, which directly affects the changes of patients' diseases. Therefore, effective sleep nursing intervention is necessary. Some researchers have found that the use of lavender essential oil and mint essential oil can help to improve the symptoms of insomnia. Therefore, as a low-risk, low-cost, low adverse reactions, and simple and easy to operate complementary therapy, aromatherapy can be used as a nondrug method for the treatment of sleep disorders, and, combined with acupoint massage, it can better solve the sleep disorder of cancer patients and improve their sleep quality.

## 4. Data and Methods

### 4.1. General Information of Patients

Sixty patients with advanced cancer admitted to a tertiary A oncology hospital in Jiangxi Province from December 2020 to March 2022 were selected. This study was randomized into trial and control groups. The control group consisted of 30 regular treatment patients and 30 regular nursing patients for advanced cancer patients, and the trial group performed a 28-day hospice care specialist nurse mediated aromatherapy based on the control group. Pain and quality of life scores were measured before and after the intervention in both groups. The experimental group consisted of 30 cases, with the mean age of 58.2 years; the control group consisted of 30 cases, with the mean age of 58.6 years;.

Inclusion criteria were as follows: cancer diagnosed by pathology or cytology, pathological stage IV, and estimated survival time ≤6 months, patient with a complaint of pain, visual analogue score ≥1, age ≥18 years old, normal sense of smell, no history of allergy to the drugs and essential oils used in this study, and the patient knowing the condition and voluntarily participating in the study and signing the informed consent form. Exclusion criteria were as follows: coma or other serious diseases, such as heart failure, renal failure, respiratory failure, liver failure, and brain metastasis, consciousness disorder or cognitive dysfunction, which is unable to cooperate with this study, discharge or death during the study period, and withdrawal from the study.

Using random number table method, 60 patients were randomly divided into test group and control group with 30 patients in each group. The grouping situation was put into an opaque envelope and the corresponding sequence number was marked on the envelope. When the subjects were included in the study, the envelopes were opened in sequence, and they were divided into different groups according to the grouping conditions in the envelopes. Different groups were arranged in different wards as far as possible. In order to avoid measurement bias, a trained nurse evaluated and collected data for all subjects, and another researcher conducted statistical analysis. This study has been reviewed and approved by the hospital ethics committee.

### 4.2. Grouping and Methods

#### 4.2.1. Grouping and Nursing Methods

The patients in the control group were given routine treatment and routine nursing. Cancer is a systemic epidemic disease. Now it is in an advanced stage and there is no way to make radical surgery. Systemic adjuvant chemotherapy can be considered. In addition, cancer patients rely on controlling the development of the disease. In order to prolong the survival time in the case of poor physical condition, patients with advanced cancer have strong pain and can be treated with powerful analgesics. In the case of poor nutrition and inability to eat, they can be treated with infusion nutrition.

On the basis of routine treatment and routine care, the patients in the observation group continued to intervene with aromatherapy mediated by hospice nurses. The aromatherapy mediated by hospice nurses is an alternative therapy that uses the pure essential oil of aromatic plants to assist medical work according to the pain grade characteristics of physical diseases of patients with advanced cancer. The role of aromatherapy is to enable patients to obtain the integrated curative effect of body, heart, and spirit. Medicinal materials with aromatic smell, such as *Angelica dahurica*, clove, frankincense, benzoin, white rosin, *Acanthopanax senticosus*, sandalwood, aloes, and musk, are made into drug types with different odors by appropriate methods. The drugs are used by burning, wearing, rubbing, or taking through the nose, mouth, and skin to penetrate into the body, improve anxiety, pain, fatigue, and other conditions, and make patients with advanced cancer happy, excited, or have mysterious feelings. It has the functions of warming the meridians, harmonizing Yin and Yang, and unblocking Qi. It has the dual functions of helping sleep and relieving pain. The personal system of patients with advanced cancer is different, which may cause skin allergy or discomfort. It is recommended to use it under the guidance of hospice nurses to avoid the side effects and contraindications of aromatherapy and drugs for cancer patients. The patients in the control group were given routine treatment and routine nursing. The patients in the observation group were given aromatherapy intervention mediated by hospice nurses on the basis of the control group. The intervention was conducted at 13:00 p.m. every day and 30 min before going to bed every night for 28 days. Before and after the intervention, the pain and quality of life of the two groups were evaluated by visual analog score and EORTC QLQ-C30.

#### 4.2.2. Statistical Methods

The clinical data were analyzed by IBM SPSS 24.0 data analysis platform. Observe the distribution law of the data, discuss the correlation between the data by using Spearman correlation analysis method, and analyze the statistical significance of the observed data by linear regression. In all data analysis, the significance *p* value of the statistical data is considered to be in the confidence space when *p* < 0.05.

## 5. Simulation Verification

### 5.1. Analysis of before and after Intervention of Two Different Therapies

Cancer can bring many uncomfortable symptoms to patients, such as pain, fatigue, anxiety, and fear. Cancer pain is considered to be one of the most common and fearful symptoms. Cancer pain is often accompanied by involvement pain in other parts. In the process of advanced treatment, most of the pain parts are not clear, and the scope is relatively broad and even covers the whole body. Pain management is based on image detection and analysis. An important part of hospice nurse mediated aromatherapy can use effective pain management techniques for patients with advanced cancer. Hospice nurses should also pay attention to educating patients about cancer pain and clarify their cognition of cancer pain, so that patients with advanced cancer can comfort themselves when they encounter pain and enhance their tolerance to pain, so as to reduce the pain of patients with advanced cancer. Now, the scores of the two groups of subjects in the total scores of sensory items, emotional items, pain, VAS, and PPI are analyzed, respectively, and Table 1 is obtained.

In Table 1, through the scoring data before and after the intervention of two different therapies in the above table, it can be clearly seen that, after the aromatherapy nursing intervention, the pain symptoms of patients with advanced cancer have been significantly improved, which also shows that aromatherapy plays a positive role in alleviating the pain of patients with advanced cancer.

In order to better observe and analyze the effects of the scores of patients with advanced cancer before and after the two different treatment interventions, the score data of patients in the above table are visualized, as shown in Figure 1.

As shown in Figure 1, the statistical results of patients with advanced cancer before and after the implementation of sensory items, emotional items, pain, VAS, and PPI are shown. The comparison between traditional therapy and aromatherapy shows that aromatherapy is significantly better than traditional therapy. It directly opened the gap between the two different therapies. Therefore, aromatherapy is worthy of application in clinical work.

### 5.2. Analysis of EORTC QLQ-C30 Score before and after Two Different Treatment Interventions

After standardized treatment, the pain symptoms of patients were relieved, especially in patients with advanced cancer. They are weakness, lack of appetite for food, fatigue, inability to take care of themselves, and other systemic symptoms. With the pain of the whole body, even the use of painkillers cannot completely relieve the pain. Most branches have metastasis and damage to adjacent organs and tissues, decreased activity tolerance, decreased physical function, and psychological anxiety, depression, and fear. With the sudden change of roles during the disease, social activities also decrease, and loneliness during hospitalization has seriously affected the quality of life of late-stage cancer patients. Now, the physical function, role function, emotional function, cognitive function, social function, fatigue, nausea, and vomiting of the two groups of subjects are analyzed, and Table 2 is obtained.

In Table 2, it can be clearly seen from the EORTC QLQ-C30 score data before and after the intervention of two different therapies in the above table that, after the nursing intervention for advanced cancer patients receiving aromatherapy, the efficacy of aromatherapy intervention can be clearly seen from the physical function and emotional function, and the degree of nausea is significantly lower than that of conventional treatment, which can directly explain that aromatherapy can reduce the incidence of nausea and vomiting.

In order to better observe and analyze the effect of EORTC QLQ-C30 score of patients with advanced cancer before and after the intervention of two different therapies, the EORTC QLQ-C30 score data of patients in the above table are visualized, as shown in Figure 2.

As shown in Figure 2, according to the visualization of EORTC QLQ-C30 score data of patients with advanced cancer, it can be clearly seen that aromatherapy can effectively improve the fatigue, nausea, and vomiting of patients with advanced cancer, so as to improve the quality of life of patients with advanced cancer.

## 6. Discussion

With the emergence of various new drugs and treatment modalities, the number of patients living with cancer is constantly increasing, but the number of patients experiencing a series of uncomfortable symptoms is also increasing, seriously affecting the quality of life of patients [14]. Pain, as one of the most common symptom burdens of cancer patients, especially late-end patients, is also a symptom with the greatest impact on patients. Moreover, the pain of cancer patients is mostly chronic pain. The World Health Organization (WHO) has listed cancer pain management as a global important issue [15]. In recent years, nondrug therapy has a positive significance in improving the pain in cancer patients, and it has the characteristics of small side effects compared with drug therapy, which is widely accepted by patients. Aromatherapy is a more common form of nonpharmacological therapy, where most of the essential oils used to improve pain are lavender and bergamot [16]. The main components of lavender essential oil are linalool, ketones, and Lin camphor ester acetate, with sedative, analgesic, and anti-inflammatory effects [17]. The main components of bergamot contain citmonene, Pineol, laurel ene, citral, and so forth, which have analgesia and pain resistance [18]. The results of this study show that the 28-day hospice care nurse-mediated aromatherapy can improve patient pain and improve patient quality of life. The difference was statistically significant (*p* < 0.05). Consistent with the results of Qian and Chen [19], Wang and Yunzi's [20] study results also showed that Aromatherapy through inhalation of lavender and bergamot essential oil can relieve the pain degree in patients with laparoscopic cholecystectomy. The mechanism of action of aromatherapy for pain relief is that essential oils enter the olfactory system through the nasal tract, and the receptor cells in the olfactory sense transmit the stimulating impulse to the limbic system of the brain. The intertwined neurons of the olfactory-limbic system enable essential oils to act on the central neuroendocrine system of the brain, which in turn can release neurotransmitters such as beta-endorphins and enkephalins, the autonomic responses to pain can be reduced and thus reduce the pain [21]. Quality of life is one of the important indicators to evaluate the treatment and rehabilitation of cancer patients. Aromatherapy alleviates the discomfort symptoms, improves bad mood, and improves sleep quality, and the aroma molecules of essential oil can stimulate the marginal system, cause patients to have happy memories of certain happy things, and then improve the quality of life [22].

Panning care specialist nurses assume the role of assessor, educator, and implementer in hospice care practice, including [23]. Nurses have the most contact with cancer patients in their clinical work, evaluate them continuously through accurate and effective evaluation tools or communication, and develop targeted interventions to relieve patients' symptoms and improve their quality of life in [24]. In the process of implementing the intervention measures, their professional ability can not only reduce the physical discomfort of the patients but also bring the psychological and spiritual dependence to the patients through the therapeutic communication. Guide patients to correctly accept the disease condition, help patients to deal with the disease well, and rebuild the purpose and meaning of life. At the same time, family members are also encouraged to actively participate in the care of patients, guide them to give patients the best comfortable care, and promote the emotional communication between patients and their families, so that they can “thank you, say love, apologize and say goodbye” at the end of their life.

## 7. Summary

In this study, based on image detection and analysis and hospice nurse mediated aromatherapy in the intelligent medical environment, the impact of pain on patients with advanced cancer was studied. Through the comparative analysis of aromatherapy and conventional therapy, using statistical methods and simulation verification, aromatherapy, as an auxiliary therapy, can achieve the purpose of improving mental state; it provides more comprehensive and accurate condition data in the nursing process of patients with advanced cancer based on image detection and analysis and hospice nurse mediated aromatherapy than conventional therapy. Image detection and analysis can make patients have a deep understanding of the condition, which is conducive to alleviate the pain of patients, relieve the discomfort of the body, and provide a good foundation for follow-up treatment. The final results showed that the effect of the observation group in pain score, QLQ-C30, value was better than that of the control group of advanced cancer patients with conventional therapy. Aromatherapy can reduce pain and muscle tension, reduce neuropathic pain scores, help to enhance self-acceptance, and cope with physical changes and improve patients' quality of life. The application of aromatherapy has a deep impact on the medical field, so that patients can improve the quality of life at the end of life, so as to further improve the core competence of hospice nurses and provide theoretical basis and practical guidance for the research and development of hospice in the future. In this study, aromatherapy based on image detection analysis and hospice care nurses in a smart medical environment is a safe, economical, and simple nonpharmacological therapy that can effectively relieve pain and improve the quality of life in cancer patients. However, there are some deficiencies in this study, and the patients' psychological mood and sleep quality were not included in the analysis. Then, the sample size will be expanded to evaluate the effect on psychological and sleep consumption.

## Figures and Tables

**Figure 1:** Visualization of simplified McGill pain questionnaire analysis.

**Figure 2:** Visualization of EORTC QLQ-C30 before and after two different treatment interventions.

**Table 1:** Simplified McGill pain questionnaire analysis.

		Total score of sensory items	Total score of emotional items	Total pain score	VAS	PPI

Before implementation	The control group	2.37 ± 1.30	7.33 ± 1.69	9.70 ± 2.37	2.47 ± 1.25	2.10 ± 0.88
	The experimental group	2.13 ± 1.61	7.10 ± 2.37	9.23 ± 3.41	2.30 ± 1.12	2.33 ± 0.92
	*t*	−0.617	−0.439	−0.616	−0.544	1
	*p*	0.54	0.662	0.54	0.589	0.321

After implementation	The control group	1.27 ± 0.52	5.90 ± 1.71	7.00 ± 1.97	1.37 ± 0.72	1.47 ± 0.53
	The experimental group	2.17 ± 0.87	7.67 ± 2.00	9.80 ± 2.23	2.07 ± 1.34	2.07 ± 0.91
	*t*	4.844	3.672	4.913	2.526	2.977
	*p*	0	0.001	0	0.014	0.004

**Table 2:** Analysis of EORTC QLQ-C30 scores before and after intervention of two different therapies.

Grouping	Somatic function	Role function	Shortness of breath	Insomnia	Loss of appetite	Nausea and vomiting	Constipation

The control group	13.11 ± 12.19	13.33 ± 14.77	74.44 ± 24.26	84.44 ± 19.04	75.56 ± 23.05	69.44 ± 17.00	80.00 ± 20.72
The experimental group	28.44 ± 27.51	31.11 ± 28.94	46.67 ± 32.28	57.78 ± 34.94	53.33 ± 33.45	47.22 ± 32.78	41.11 ± 39.81
*t*	−1.889	−2.417	−3.425	−3.094	−2.676	−2.691	−3.78
*p*	0.059	0.016	0.001	0.002	0.007	0.007	0

## Data Availability

The data underlying the results presented in the study are available within the manuscript.
